# Effect of Wnt Signaling on the Differentiation of Islet *β*-Cells from Adipose-Derived Stem Cells

**DOI:** 10.1155/2017/2501578

**Published:** 2017-02-20

**Authors:** Hefei Wang, Yu Ren, Xiao Hu, Min Ma, Xiao Wang, Hao Liang, Dongjun Liu

**Affiliations:** ^1^National Research Center for Animal Transgenic Biotechnology, Inner Mongolia University, Hohhot, Inner Mongolia 010070, China; ^2^Laboratory for Reproductive Health, Institute of Biomedicine and Biotechnology, Shenzhen Institute of Advanced Technology, Chinese Academy of Sciences, Shenzhen, Guangdong 518055, China

## Abstract

The Wnt signaling is critical for pancreatic development and islet function; however, its precise effects on the development and function of the *β*-cells remain controversial. Here we examined mRNA and protein expression of components of the Wnt signaling throughout the differentiation of islet *β*-cells from adipose-derived stem cells (ADSCs). After induction, ADSCs expressed markers of *β*-cells, including the* insulin*,* PDX1*, and* glucagon* genes, and the PDX1, CK19, nestin, insulin, and C-peptide proteins, indicating their successful differentiation. Compared with pancreatic adult stem cells (PASCs), the quantities of* insulin*,* GLUT2*, and* Irs2* mRNA decreased, whereas* Gcg*,* Gck*,* and Irs1* mRNA increased. Over time, during differentiation,* insulin* mRNA and protein expression increased,* Gcg* and* Gck* mRNA expression increased,* Irs1* mRNA expression decreased and then increased, and* Irs2* mRNA increased and then decreased (all *P* < 0.05). The expression of* Dvl-2*,* LRP5*, and* GSK3β* mRNA as well as the Dvl-2, GSK3*β*, and p-GSK3*β* proteins also increased (*P* < 0.05). Expression of* TCF7L2* (6–10 d) and *β-catenin* mRNA as well as the *β*-catenin protein increased but not significantly (*P* > 0.05). Our results indicate that the Wnt signaling is activated during ADSC differentiation into islet *β*-cells, but there was no obvious enrichment of nonphosphorylated *β*-catenin protein.

## 1. Introduction

Adipose-derived stem cells (ADSCs) can differentiate into multiple cell types [1] and offer many advantages for tissue engineering and transplantation [2–4], such as easy acquisition, high yield, and low immunogenicity [5–7]. In a previous study, human ADSCs were differentiated into insulin-producing cells (IPCs) and transplanted into the mouse model of type 2 diabetes mellitus (T2DM), resulting in an increased level of circulating insulin and a subsequent improvement in metabolic parameters and blood glucose reduction [8]. Therefore, investigating the mechanisms behind the differentiation of ADSCs into islet *β*-cells is required to confirm their efficiency in the therapy of T1DM and T2DM.

The Wnt/*β*-catenin signaling pathway regulates and controls the growth, differentiation, and translocation of cells [9] and is critical for the development of the pancreas, islet function, and the generation and secretion of insulin [10]. *β*-Catenin (which activates the expression of target genes [11, 12]) has been shown to elicit different effects throughout the different developmental phases of the pancreas [13]. For example, *β*-catenin promotes fibroblast growth factor (FGF) expression and Hedgehog signaling and hinders pancreatic duodenal homeobox-1 (PDX1) expression in the early phase of the development of the pancreas and promotes proliferation of the pancreatic cells and growth of the pancreas in the late phase. Furthermore, after the Wnt pathway, activator (Wnt-3a) or *β*-catenin protein was added to *β*-cells or pancreatic islets in culture, expression of PITX2 (a direct target of Wnt signaling) and Cyclin D2 (an important regulator of the *β*-cell cycle) was promoted, *β*-cells were proliferated, and serum insulin increased in vitro [14]. However, after adding Axin (a negative regulator of the Wnt pathway), expression of PITX2 and Cyclin D2 was reduced, the number of *β*-cell clusters decreased, and glucose tolerance was damaged [14]. Moreover, silencing of the T-cell factor 7-like 2 (TCF7L2) (an important transcription factor of the Wnt/*β*-catenin signaling pathway) gene increased the apoptosis of pancreatic *β*-cells, reduced *β*-cell proliferation, and, thereby, reduced insulin secretion [15]. Indeed, the loss of insulin secretion due to the loss of function of TCF7L2 in the pancreatic islet and polymorphisms of the human* TCF7L2* allele further indicate that the susceptibility and pathogenesis of diabetes mellitus may be caused by disturbance of the Wnt signaling pathway [16]. While the roles of *β*-catenin/TCF7L2 in pancreatic development, islet function, and generation and secretion of insulin have been determined, the effects of the Wnt/*β*-catenin signaling pathway on the development and function of the endocrine cells of the pancreatic islet (including the *β*-cells generating insulin) remain controversial [17].

Therefore, in this study, we induced the differentiation of ADSCs into insulin-producing cells and monitored the changes in the Wnt/*β*-catenin signaling pathway components and related factors at a transcriptional and translational level over time. The aim of our study was to confirm the role of the Wnt/*β*-catenin signaling pathway in the development and function of pancreatic *β*-cells generating insulin.

## 2. Materials and Methods

### 2.1. Reagents

Low glucose Dulbecco's modified Eagle's medium (DMEM) (10567-014) and DMEM containing 4.5 g/L glucose (11965-092) were purchased from Gibco-BRL (Gaithersburg, MD). Dithizone (D5130) was from Sigma (St. Louis, MO). DMSO (042-21765) was from Wako (Tokyo, Japan). Recombinant human DKK-1 (5439-DK-010) and recombinant human Wnt-3a (5036-WN-010) was from R&D Inc. (Minneapolis, MN). Insulin antibody (sc-9168) was from Santa Cruz Biotechnology (Dallas, TX). C-peptide (ab14181) and GSK3*β* (ab93926) antibodies were from Abcam (Cambridge, UK). Phospho-GSK3*β* (Ser9) (D3A4) (9322S), non-phospho- (active) *β*-catenin (Ser33/37/Thr41) (D13A1) (8814S), and Dvl-2 (30D2) (3224P) antibodies were from Cell Signaling Technology (Beverly, MA). CD13 (BA0718), CD44 (BA0321), CD106 (BA0406), and CD49d (BA1640) antibodies were from Boster Biological (Wuhan, China). Pancreatic and duodenal homeobox-1 (PDX1, bs-0923R) antibody was from Bioss (Beijing, China). Cytokeratin 19 (CK19, BA2266) and nestin (BA1289) antibodies were from Boster Biological (Wuhan, China).

### 2.2. Animals

Wistar rats (aged 5-6 weeks) were purchased from the National Research Center for Animal Transgenic Biotechnology, Inner Mongolia University. All studies adhered to procedures consistent with the National Research Council Guide for the Care and Use of Laboratory Animals and were approved by the Institutional Animal Care and Use Committee of Inner Mongolia University. All rat treatments were performed with efforts to minimize suffering and rats were killed by cervical dislocation.

### 2.3. Isolation, Culture, and Identification of Rat ADSCs

The epididymal fat from male Wistar rats aged 5-6 weeks was obtained under aseptic conditions. ADSCs were then isolated and cultured according to our previous method [18]. Surface markers of passage 3 (P3) ADSCs were detected immunohistochemically using CD13 (1 : 300), CD44 (1 : 300), CD106 (1 : 300), and CD49d (1 : 300) antibodies and visualized under a confocal microscope (A1R, Nikon, Tokyo, Japan). Cell morphology was monitored using an inverted microscope (Observer A1, Zeiss, Oberkochen, Germany).

### 2.4. Isolation, Culture, and Identification of Rat Pancreatic Adult Stem Cells (PASCs)

Pancreatic tissue was harvested from Wistar rats aged 5-6 weeks under aseptic conditions. PASCs were then isolated and cultured as described previously [18]. Cell surface markers of P3 PASCs were detected immunohistochemically using PDX1 (1 : 300), CK19 (1 : 300), nestin (1 : 300), and insulin (1 : 300) antibodies. Cytokeratin 19 (CK19) [19] and nestin [20] are markers of PASCs, insulin is an important hormone generated by islet *β*-cells, and PDX1 is essential for maintaining the normal function of pancreatic islets.

### 2.5. Induction and Detection of Islet *β*-Cells

ADSCs were cultured at P3–P5 to reach ~80%–90% confluence and then induced to differentiate in DMEM low glucose culture medium containing 1% DMSO for 3 days. Complete induction of islet *β*-cell differentiation was then performed using 4.5 g/L D-glucose DMEM culture medium containing 10% FBS for 7 days. The process of induction was conducted at 37°C in 5% CO_2_ and saturated humidity. After induction, cells were dyed for 30 min at 37°C with the addition of 10 mg/mL dithizone stock solution to the culture medium at a dilution of 1 : 100. After discarding the culture medium, cells were washed three times with PBS and observed under the microscope. Then, cell surface markers of islet *β*-cells were detected immunohistochemically using the following four antibodies: PDX1, CK19, nestin, and insulin. Reverse-transcription (RT) PCR identification of islet *β*-cells was conducted using a commercial kit (TaKaRa, Dalian, China) and all PCR primers (Table 1) were synthesized by TaKaRa. The PCR reaction was as follows: 94°C for 4 min for predenaturing, followed by 43 cycles of 94°C for 5 s, 52°C for 5 s, and 72°C for 10 s and a final extension at 72°C for 5 min.

### 2.6. Quantitative PCR

The mRNA levels of genes relating to insulin secretion, as well as islet *β*-cell growth and function, were analyzed by quantitative PCR (qPCR). Specific primer pairs (cross-intron) were designed based on the mRNA sequences of* Rattus norvegicus* (provided by NCBI) for* insulin*,* glucagon (Gcg)*,* glucokinase (Gck)*,* glucose transporter type 2 (GLUT2)*,* insulin receptor substrate 1 (Irs1)*, and* insulin receptor substrate 2 (Irs2)* and synthesized by TaKaRa (Table 2). The relative difference in gene expression was calculated using the 2^−ΔΔCt^ method. The mRNA levels from PASCs were used as normal calibration samples and ADSCs induced into insulin-producing cells were used as the experimental samples. The qPCR was performed using a 7500 Real-Time PCR System (Applied Biosystems) using the following conditions: 95°C for 30 s and 50 cycles of 95°C for 5 s and 60°C for 34 s.

### 2.7. Western Blotting

Protein concentrations were measured using the BCA method after extracting the total protein from the insulin-producing cells induced from ADSCs. The total protein from PASCs was used as a reference. Proteins (45 *μ*g total) were added to each well of a SDS-polyacrylamide gel and separated by electrophoresis. Insulin and C-peptide antibodies were diluted at 1 : 500 and 1 : 100, respectively. Antibody binding was visualized using the ECL chemiluminescence reaction and the Tanon 5200 instrument. The difference in insulin and C-peptide protein expression was determined using ImageJ software.

### 2.8. Molecular Signals Involved in Induction of Islet *β*-Cells

During the induction of islet *β*-cells from ADSCs, we added Wnt-3a (an activator of Wnt signaling) or DKK-1 (an inhibitor of Wnt signaling) to the culture medium (final concentration of 100 ng/mL) and cultivated the cells for 3, 6, and 10 days to monitor the changes in the Wnt signaling pathway over time. The mRNA levels of genes relating to Wnt signaling were analyzed by qPCR. Specific primer pairs (cross-intron) were designed based on the mRNA sequences of* R. norvegicus* (provided by NCBI) for* dishevelled 2 (Dvl-2)*,* low-density lipoprotein receptor-related protein 5 (LRP5)*,* glycogen synthase kinase 3 beta (GSK3β)*, *β-catenin*, and* TCF7L2* and synthesized by TaKaRa (Table 3). The mRNA levels of related genes in the ADSCs cultured in the DMEM low glucose culture medium containing 1% DMSO for 3 days were used as a normal calibration sample.

Total protein was isolated from the insulin-producing cells induced from ADSCs over time. The samples were labeled L3, H3, and H7 in the islet *β*-cell induced media alone at 3, 6, and 10 days, labeled W-L3, W-H3, and W-H7 in the islet *β*-cell induced media with Wnt-3a at 3, 6, and 10 days, and labeled D-L3, D-H3, and D-H7 in the islet *β*-cell induced media with DKK-1 at 3, 6, and 10 days. The primary antibodies used for Western blotting were Dvl-2 (1 : 1000), non-phospho- (active) *β*-catenin (Ser33/37/Thr41) (non-p-*β*-cat) (1 : 1000), GSK3*β* (1 : 1000), phospho-GSK3*β* (Ser9) (p-GSK3*β*, Ser9) (1 : 1000), and insulin (1 : 500). Insulin levels in insulin-producing cells induced from ADSCs at different time points were also detected by immunostaining (insulin antibody diluted at 1 : 300). Stained cells were observed by confocal microscopy (A1R, Nikon, Tokyo, Japan).

### 2.9. Statistical Analysis

All data are the result of at least three independent experiments and are indicated by the mean ± standard deviation. Data were analyzed using SPSS 17.0 software (IBM Corporation, USA). The least significant difference (LSD) method was applied for comparison among groups, with *P* < 0.05 indicating statistical significance.

## 3. Results

### 3.1. Morphological Characteristics of ADSCs

Parts of the cells started to adhere to the wall when the ADSCs were subjected to inoculation for 4–6 h. They had a small circle or short stick-like shape and were unequal in size. ADSCs gradually expanded into spindles or irregular polygons after 48 h. They presented as fibroblast-like after 3 days and reached 80%–90% confluence after 6-7 days. After subculturing, ADSCs presented as gyrate or parallel spindle-shaped adherent cells, which grew densely (Figures 1(a)–1(c)).

### 3.2. Morphological Characteristics of PASCs

After digestion with collagenase V, some cell aggregates and single scattered cells were present in the cell suspension. After being cultivated for 60 h, the single cells adhered to the wall and were short and spindle-shaped in appearance. After replacing the DMEM no glucose culture medium containing 0.5% of FBS 2 weeks later for screening and purification, the majority of the cells were dead. Residual cells became proliferative after 4 days in the culture medium containing basic FGF (bFGF), and subculturing was required every 5-6 days. Subcultured PASCs were dense and fusiform or cobblestone-like in appearance (Figures 1(g)–1(i)).

### 3.3. Morphological Characteristics of Insulin-Producing Cells

No obvious changes were observed when ADSCs were subjected to induction for 3 days in DMEM low glucose culture medium containing 1% DMSO and still presented as spindles or polygons, with clear cell nuclei. However, the cells started to aggregate when ADSCs were subjected to induction for 3 days in 4.5 g/L D-glucose DMEM culture medium containing 10% FBS. The cells grew densely after being induced for 5 days, with circular clusters and significantly increased refractivity. After 7 days, the majority of ADSCs formed clusters (Figures 1(d)–1(f)).

### 3.4. Identification of Surface Markers of ADSCs and PASCs

The surface markers of CD13, CD44, and CD49d in the ADSCs were positive. CD13 showed weak expression, CD49d showed strong expression, and CD106 showed little expression (Figures 2(a)–2(e)). These results are in line with literature reports [5, 21–23] and indicate that pure ADSCs were acquired by digestion with type I collagenase and then adherent cultivation. Similarly, the surface markers PDX1, nestin, CK19, and insulin in the PASCs were positive, indicating that PASCs were acquired successfully by separation (Figures 2(k)–2(o)).

### 3.5. Induction of Insulin-Producing Cells

After induction of rat ADSCs into insulin-producing cells, the majority of the cell clusters were brown/red after dyeing with dithizone, indicating that zinc ions were rich in the cytoplasm, proving the presence of insulin-producing cells (IPCs) (Figure 3(a)). The majority of PASCs were also dyed brown/red (Figure 3(b)), while ADSCs were not (Figure 3(c)).

Positive expression of PDX1, nestin, CK19, and insulin was observed in the ADSCs induced into insulin-producing cells. (Figures 2(f)–2(j)). These results indicate that the ADSCs had successfully transdifferentiated into insulin-producing cells. Similarly, expressions of* GAPDH*,* insulin*,* PDX1*, and* glucagon* genes were detected in the insulin-producing cells induced from ADSCs (Figure 4(C)).* GAPDH*,* insulin*, and* PDX1* genes were also detected in PASCs, while no* glucagon* gene was detected (Figure 4(B)). Only* GAPDH* was expressed in the ADSCs after common cultivation (Figure 4(A)). Therefore,* insulin* and* PDX1* of PASCs are expressed in insulin-producing cells induced from ADSCs; however, unlike the PASCs,* glucagon* was also expressed in insulin-producing cells induced from ADSCs.

### 3.6. Differential mRNA Expression between PASCs and Insulin-Producing Cells

Quantitative PCR analysis indicated that the mRNA expression quantities of* insulin*,* Gcg*,* Gck*,* GLUT2*,* Irs1*, and* Irs2* in insulin-producing cells induced from ADSCs were 0.69 times (*P* < 0.05), 2.12 times (*P* < 0.01), 1.15 times (*P* > 0.05), 0.58 times (*P* < 0.01), 1.38 times (*P* < 0.01), and 0.83 times (*P* < 0.01) those in PASCs, respectively (Figure 5). GLUT2 regulates the synthesis and secretion of insulin and is specifically expressed on the membrane of islet *β*-cells. Together with Gck, GLUT2 forms the glucose sensor that facilitates the entrance of glucose into the cell. Gck senses the concentration of glucose in the *β*-cell and is an important downstream target gene of the classical Wnt signaling pathway. Irs1 and Irs2 are two substrate proteins related to *β*-cell function.

### 3.7. Differential Protein Expression between PASCs and Insulin-Producing Cells

Expressions of insulin and C-peptide protein differed between PASCs and insulin-producing cells induced from ADSCs, with the relative expression of insulin and C-peptide in insulin-producing cells induced from ADSCs being lower than that in the PASCs (Figure 6).

### 3.8. Molecular Signals Involved in the Induction of Insulin-Producing Cells from ADSCs

Insulin mRNA and protein expression increased (*P* < 0.01) during the induction of insulin-producing cells from ADSCs. In addition,* Gcg* and* Gck* mRNA expression increased (*P* < 0.05), while* Irs1* mRNA expression decreased and then increased (*P* < 0.01), and* Irs2* mRNA expression increased and then decreased (*P* < 0.01).* Dvl-2*,* LRP5*, and* GSK3β* mRNA expression also increased (*P* < 0.05) during the induction of insulin-producing cells from ADSCs over time. While the expression of *β-catenin* mRNA increased, the change was not statistically significant (*P* > 0.05). Similarly, the expression of* TCF7L2* mRNA increased from day 6 to day 10 but not significantly (*P* > 0.05). Correspondingly, Dvl-2, GSK3*β*, and p-GSK3*β* protein expressions significantly increased (*P* < 0.01), while non-p-*β*-catenin protein expression did not (*P* > 0.05). Therefore, although the Wnt signaling pathway was activated, enrichment of the nonphosphorylated *β*-catenin protein was not obvious during the differentiation of ADSCs into the insulin-producing cells by DMSO and a high content of glucose.

When the activator of the Wnt signaling pathway (Wnt-3a) was added, Dvl-2 mRNA and protein expression increased transitorily on day 3,* LRP5* mRNA expression increased on day 10, GSK3*β* mRNA and protein expression increased on day 6, p-GSK3*β* protein expression increased on day 6, *β*-catenin mRNA expression increased with time (but protein expression did not), and TCF7L2 mRNA expression increased on day 3. Correspondingly, insulin mRNA and protein expression increased gradually after adding Wnt-3a; Gcg and Gck mRNA expression increased during this period; and GLUT2 mRNA expression increased obviously on day 10. When the inhibitor of the Wnt signaling pathway (DKK-1) was added, Dvl-2 mRNA and protein expression decreased, LRP5 mRNA expression decreased on day 6, GSK3*β* mRNA and protein expression decreased on day 10, p-GSK3*β* protein expression decreased on day 10, non-p-*β*-catenin protein expression decreased on day 10, and TCF7L2 mRNA expression decreased on day 6. Correspondingly, insulin protein expression decreased gradually after adding DKK-1 (Figures 7 and 8).

Consistent with the Western blot analysis, insulin protein expression increased over time when examined immunohistochemically (Figures 9(a), 9(e), and 9(i)). Insulin expression also increased from day 3 to day 10 in the presence of Wnt-3a (Figures 9(b), 9(f), and 9(j)) but decreased in the presence of DKK-1 (Figures 9(c), 9(g), and 9(k)). Insulin protein expression increased after activating the Wnt pathway, and its expression in the later phase (i.e., at day 10) could be decreased by blocking the Wnt pathway during the induction of insulin-producing cells from ADSCs.

## 4. Discussion

In this study, we examined changes in the mRNA and protein expression of components of the Wnt signaling pathway when ADSCs were inducted to differentiate into islet *β*-cells. We confirmed that ADSCs could be induced to differentiate into insulin-producing cells using DMSO and a high glucose condition [24]. The expressions of PDX1, CK19, nestin, and insulin proteins (as well as the corresponding marker genes) were in line with the results of previous studies, indicating that the ADSCs had differentiated toward islet *β*-cells. Moreover, our results with the Wnt activator and inhibitor indicate that the Wnt signaling pathway may be important for this differentiation process. Therefore, our study provides evidence for the role of the Wnt/*β*-catenin signaling pathway in the differentiation of pancreatic *β*-cells generating insulin from ADSCs.

The expression of PDX1 protein observed in this study provides further evidence for its role in the differentiation of pancreatic *β*-cells. PDX1 has previously been shown to be the crucial transcriptional factor involved in the differentiation and development of pancreatic islet cells [25]. Indeed, human ADSCs transfected with the* PDX1* gene show increased secretion of glucose-stimulated insulin, indicating that hADSCs were induced to differentiate into IPCs by the expression of exogenous PDX1 [26]. Moreover, overexpression of PDX1 by lentivirus in hADSCs induces their differentiation into insulin-producing cells, which, in turn, secrete insulin [27]. Therefore, the differentiation of ADSCs into pancreatic insulin-producing cells by PDX1 offers a potential strategy for *β*-cell replacement therapy in T1DM.

The induction method in the current study was relatively economical, simple, and quick; however, different in vitro induction methods have been used previously for the differentiation of mesenchymal stem cells (MSCs) into islet cells [28, 29]. A previous study showed that MSCs could generate IPCs using mouse neonate pancreas extract, by expressing genes related to *β*-cells (*PDX1*,* INS1*,* INS2*,* EP300*, and* CREB1*), and found a dialogue between the FOXA2 and TCF7L2 transcription factors [30]. Moreover, the DNA-PK compound and KAT2B were shown to interact with PDX1, CREB1, and EP300, leading to the induction of IPCs and generation of insulin [30]. Therefore, our induction method might be further perfected by introducing certain genes regulating the development of the pancreas islet into ADSCs [31] and then detecting the quantity of the insulin secretion outside the cell.

While the classical Wnt/*β*-catenin is known to play a role in the development and function of insulin producing *β*-cells, its precise function remains controversial [17]. In this pathway, the Wnt ligand combines with the Frizzled (Fz) and LRP5/6 receptors. Fz then recruits Dvl, leading to phosphorylation at the LRP5/6 intracellular terminal. Axin is recruited to the cytomembrane nearby, thereby preventing *β*-catenin from being degraded by complexes composed of Axin, GSK3, APC, and CK1, among others. Without Wnt ligand stimulation, *β*-catenin is phosphorylated and degraded by the proteasome. In the current study, we found that the expression of Dvl-2, GSK3*β*, and p-GSK3*β* proteins increased during differentiation of ADSCs into insulin-producing cells over time, indicating that the Wnt signaling pathway was activated. However, we found no obvious enrichment of the nonphosphorylated *β*-catenin protein. Indeed, Baumgartner et al. [32] recently stated that the effect of *β*-catenin on the development of *β*-cells is controversial. The number of *β*-cell clusters decreased as a result of specific deletion of *β*-catenin in the pancreas, which correlated with an early and specific loss of multipotent pancreatic progenitor cells [32]. Murtaugh et al. [33] also showed that if the *β*-catenin gene was deleted, the pancreas became hypoplastic, but the function of the islet endocrine cell mass was not significantly perturbed. Furthermore, Keefe et al. [34] proved that *β*-catenin is continuously required for the establishment and maintenance of the pancreatic acinar cell mass, but this requirement is not shared with islet cells, which can proliferate and function normally in the absence of *β*-catenin. Therefore, loss of Wnt/*β*-catenin activity is unlikely to drive islet dysfunction. In this study, we found that *β*-catenin mRNA expression increased over time when the Wnt-3a activator of the Wnt signaling pathway was added; however, the *β*-catenin protein expression did not change obviously. Despite this, the expression quantities of insulin mRNA and protein increased gradually when Wnt-3a was added. Therefore, our study provides further evidence that the Wnt signaling pathway is activated during differentiation of ADSCs into insulin-producing cells and promotes the expression of insulin over time, as summarized in Figure 10.

To date, studies of the Wnt/*β*-catenin signaling pathway have focused on osteoblast differentiation of stem cells, and the results remain disputed. D'Alimonte et al. [35] showed that the canonical Wnt/*β*-catenin signaling pathway might trigger osteoblast differentiation of human amniotic fluid MSCs, and the expressions of Dvl-2, nonphosphorylated *β*-catenin, and p-GSK3*β*^Serine9^ increased in the early stage of osteoblast differentiation. However, Cho et al. [36] reported that the endogenous Wnt signal could promote proliferation of ADSCs and restrain osteoblast differentiation. Therefore, using RNAi of the Wnt signal should restrain the expression of *β*-catenin and promote osteoblast differentiation of ADSCs. Furthermore, treatment with Wnt-3a conditioned media increased cellular *β*-catenin levels and the rate of cellular proliferation but inhibited osteogenic differentiation [36]. Therefore, the role of the Wnt/*β*-catenin signaling pathway should be further studied with respect to stem cell differentiation, as different differentiation effects may occur in different types of stem cells.

In conclusion, this study confirmed the positive effect of the Wnt signaling pathway on the differentiation of insulin-producing cells from ADSCs. After analyzing the gene expression profiles at three different stages (adhesion, expansion, and differentiation) during in vitro islet generation, Dodge et al. [37] showed that the expression of insulin, glucagon, duct markers (mucin 6 and aquaporin 1 and 5), and the *β*-cell autoantigen IA-2/phogrin increased in the differentiation stage. In addition, developmentally important pathways including notch/jagged, Wnt/frizzled, TGF*β* superfamily (follistatin, BMPs, and SMADs) and retinoic acid (COUP-TFI, CRABP1, 2, and RAIG1) were differentially regulated during the expansion/differentiation stage [37]. Therefore, in the future, appropriate manipulation of these differentiation-associated pathways will enhance the efficiency of differentiation of islet *β*-cells in vitro for the use in treatment of diseases such as T1DM and T2DM.

## Figures and Tables

**Figure 1:** Morphology of rat ADSCs, rat ADSCs induced into insulin-producing cells, and rat PASCs (100x). (a–c) Recently detached, primary, and passage 11 rat ADSCs. (d–f) Preinduction rat ADSCs, ADSCs induced with DMEM low glucose containing 1% DMSO after 3 days, and ADSCs induced with 4.5 g/L D-glucose DMEM containing 10% FBS to differentiate into insulin-producing cells after 7 days. (g–i) Recently detached rat PASCs, PASCs purified with DMEM no glucose containing 0.5% FBS after 2 weeks, and P3 PASCs cultured with DMEM low glucose containing basic fibroblast growth factor (bFGF).

**Figure 2:** Immunostaining of rat ADSCs, rat ADSCs induced into insulin-producing cells, and rat PASCs. (a–e) CD13, CD44, CD49d, CD106, and control group (no primary antibody) staining of rat ADSCs. (f–j) PDX1, nestin, CK19, insulin, and control group staining of rat ADSCs induced into insulin-producing cells. (k–o) PDX1, nestin, CK19, insulin, and control group staining of rat PASCs. Magnification: ×100.

**Figure 3:** Dithizone staining (100x) of (a) ADSCs induced into insulin-producing cells, (b) rat PASCs, and (c) rat ADSCs.

**Figure 4:** Electrophoresis of the RT-PCR products of (A) rat ADSCs, (B) rat PASCs, and (C) rat ADSCs induced into insulin-producing cells.

**Figure 5:** Differential mRNA expression in rat ADSCs induced into insulin-producing cells compared with rat PASCs as determined by quantitative PCR. Data are presented as the mean ± standard deviation. ^*∗*^*P* < 0.05 and ^*∗∗*^*P* < 0.01, compared with rat PASCs.

**Figure 6:** Comparison of protein expression levels of insulin (H-86) and C-peptide in (A) rat ADSCs induced into insulin-producing cells and (B) rat PASCs. Data are presented as the mean ± standard deviation. ^*∗*^*P* < 0.05 and ^*∗∗*^*P* < 0.01, compared with rat PASCs.

**Figure 7:** (a)* Dvl-2*, (b)* LRP5*, (c)* GSK3β*, (d) *β-catenin*, (e)* TCF7L2*, (f)* insulin*, (g)* Gcg*, (h)* Gck*, (i)* GLUT2*, (j)* Irs1*, and (k)* Irs2* mRNA expression in rat ADSCs induced into insulin-producing cells over time by real-time PCR. Data are presented as the mean ± standard deviation. ^*∗*^*P* < 0.05 and ^*∗∗*^*P* < 0.01, compared with L3 (ADSCs cultured in the DMEM low glucose culture medium containing 1% DMSO for 3 days).

**Figure 8:** Western blot analysis of relative levels of insulin and Wnt pathway protein expression in rat ADSCs induced into insulin-producing cells over time (L3, H3, and H7) and in the presence of the Wnt-3a activator (W-L3, W-H3, and W-H7) or the DKK-1 inhibitor (D-L3, DH3, and D-H7). Data are presented as the mean ± standard deviation. ^*∗*^*P* < 0.05 and ^*∗∗*^*P* < 0.01, compared with L3 (ADSCs cultured in the DMEM low glucose culture medium containing 1% DMSO for 3 days).

**Figure 9:** Immunofluorescence staining of insulin in rat ADSCs induced into insulin-producing cells over time. (a–d) Induction into insulin-producing cells (L3), addition of Wnt-3a (W-L3), addition of DKK-1 (D-L3) for 3 days, and control group of rat ADSCs. (e–h) Induction into insulin-producing cells (H3), addition of Wnt-3a (W-H3), addition of DKK-1 (D-H3) for 6 days, and control group of rat ADSCs. (i–l) Induction into insulin-producing cells (H7), addition of Wnt-3a (W-H7), addition of DKK-1 (D-H7) for 10 days, and control group of rat ADSCs. Magnification: ×100.

**Figure 10:** Schematic diagram depicting proposed mechanism for the Wnt signaling pathway activation during differentiation of ADSCs into insulin-producing cells. ADSCs, in the induction of islet *β*-cells medium, initiate islet *β*-cells differentiation. Islet *β*-cells commitment is linked to the stimulation of the canonical Wnt pathway that sequentially involves the following: the Wnt ligand combines with the Frizzled (Fz) and LRP5/6 receptors. Fz then recruits Dvl, leading to phosphorylation at the LRP5/6 intracellular terminal. The phosphorylation of GSK3*β* leads to the inactivation of a cytoplasmic complex composed of CK1, Axin, APC, and GSK3*β* and detachment of *β*-catenin phosphorylation from the complex. These events result in the increase of *β*-catenin mRNA, but it was not obvious in *β*-catenin protein (possibly undergoing posttranscriptional modifications, actions of miRNA, etc.). The *β*-catenin stabilization activates the islet *β*-cells marker insulin in the transcriptional and translational levels. DKK-1 is a secreted Wnt antagonist that may be used as a drug to inhibit Wnt signal. CK1, casein kinase 1; DKK-1, Dickkopf 1; Dvl, dishevelled; GSK3*β*, glycogen synthase kinase 3*β*; LRP5/6, low-density lipoprotein receptor-related protein 5/6; TCF, T-cell factor.

**Table 1:** Primers used for RT-PCR identification of islet *β*-cells.

Primer name	Primer sequence (5′-3′)	Size (bp)
GAPDH	Forward: TGAACGGGAAGCTCACTGG	360
	Reverse: TCCACCACCCTGTTGCTGTA	
Insulin	Forward: TACAATCATAGACCATCAGCA	235
	Reverse: CAGTTGGTAGAGGGAGCAGAT	
PDX1	Forward: TACAAGCTCGCTGGGATCACT	268
	Reverse: GCAGTACGGGTCCTCTTGTT	
Glucagon	Forward: GACCGTTTACATCGTGGCGG	199
	Reverse: CGGTTCCTCTTGGTGTTCATCAAC	

**Table 2:** Primers used for quantitative PCR analysis of islet *β*-cell growth and function genes.

Primer name	Primer sequence (5′-3′)	Size (bp)
GAPDH	Forward: GGCACAGTCAAGGCTGAGAATG	143
	Reverse: ATGGTGGTGAAGACGCCAGTA	
Insulin	Forward: AGCGTGGCATTGTGGATCAG	117
	Reverse: TCAAAGGCTTTATTCATTGCAGAGG	
Gcg	Forward: ACTGGCTGATTCAAACCAAGATCAC	150
	Reverse: ATGTATTCGTCCGCATGCAAAG	
Gck	Forward: AGTATGACCGGATGGTGGATGAA	114
	Reverse: CCAGCTTAAGCAGCACAAGTCGTA	
GLUT2	Forward: GACCGGCACATGCTCTCATC	102
	Reverse: TTGGAGCAATCTCGCCAATGTA	
Irs1	Forward: AAGCACCTATGCCAGCATCAAC	106
	Reverse: GAGGATTGCTGAGGTCATTTAGGTC	
Irs2	Forward: TCTGCCAGCACCTACGCAAG	159
	Reverse: TGAGCAGCGTTGGTTGGAA	

**Table 3:** Primers used for quantitative PCR analysis of Wnt signaling pathway genes.

Primer name	Primer sequence (5′-3′)	Size (bp)
Dvl-2	Forward: CATGAGCAATGACGATGCTGTG	151
	Reverse: AGCTGGATCAATTGGCTGTATGG	
LRP5	Forward: ACCATTGATTACGCCGACCAG	141
	Reverse: ATCGCTATATTGAGTCAGGCCAAAG	
GSK3*β*	Forward: TTCTCGGTACTACAGGGCACCA	107
	Reverse: GTCCTAGCAACAATTCAGCCAACA	
*β*-Catenin	Forward: GTCTGAGGACAAGCCACAGGACTAC	115
	Reverse: AATGTCCAGTCCGAGATCAGCA	
TCF7L2	Forward: TGTGTACCCAATCACGACAGGAG	127
	Reverse: GATTCCGGTCGTGTGCAGAG	
